# Clinical Efficacy of Carbon Dioxide Laser Combined with ALA Photodynamics in the Treatment of Condyloma Acuminatum

This article has been retracted.

**DOI:** 10.1155/2021/7211055

**Published:** 2021-10-18

**Authors:** Chunyu Cao, Lihua Chen, Shu Li, Lili Yuan, Yishan Wang

**Affiliations:** Department of Dermatology, Taizhou Clinical Medical School of Nanjing Medical University (Taizhou People's Hospital), Taizhou 225300, Jiangsu, China

## Abstract

'*Purpose*. To observe the clinical efficacy and safety of carbon dioxide laser combined with ALA photodynamics in the treatment of condyloma acuminatum. *Method*. A total of 211 patients with condyloma acuminatum admitted to our hospital from April 2018 to June 2021 were selected as the observation object. They were divided into the intervention group (CO_2_ laser combined with ALA photodynamic therapy, 125 cases) and conventional group (CO_2_ laser treatment, 86 cases), and the efficacy and incidence of adverse reactions between the two groups were compared. *Result*. The total effective rate of the intervention group (96.00%) was significantly higher than that of the conventional group (84.88%) (*P* < 0.05). The total incidence of adverse reactions in the intervention group (8.00%) was lower than that in the conventional group (32.56%) (*P* < 0.05). Univariate analysis showed that the patient's smoking history, drinking history, course of disease, wart area, and number of sexual partners were related to the short-term prognosis (*P* < 0.05). Multivariate logistic regression analysis showed that the patient's course of disease, the area of the wart body, and the number of sexual partners were independent factors affecting the prognosis of patients with condyloma acuminatum (*P* < 0.05). *Conclusion*. Carbon dioxide laser combined with ALA dynamics treatment of condyloma acuminatum significantly improves the clinical efficacy, does not increase the incidence of adverse reactions, and has important clinical therapeutic value. The course of the disease, the area of the wart, and the number of sexual partners are independent factors affecting the prognosis of patients with condyloma acuminatum.

## 1. Introduction

Condyloma acuminata (CA) is a common sexually transmitted disease caused by human papillomavirus infection. It is mainly manifested in proliferative damage of anus and genitalia. With changes in lifestyle and social concepts, the incidence rate has increased significantly, which has a serious impact on the health and quality of life of patients [1, 2]. Carbon dioxide laser is an important method for the treatment of CA. It can output invisible infrared laser, which is characterized by fine beam and high energy density. It is used to burn away condyloma acuminatum to achieve the purpose of treatment [3, 4]. ALA photodynamics is a new method for the treatment of skin diseases in the clinic. It uses photosensitive drugs and laser activation treatment principles to destroy the focal tissue [5, 6]. This study mainly explores the clinical efficacy and safety of the carbon dioxide laser combined with ALA photodynamics in the treatment of CA. The report is as follows.

## 2. Materials and Methods

### 2.1. General Information

A total of 211 patients with CA diagnosed and treated in our hospital from April 2016 to June 2018 were selected as observation objects. Among them, 113 were males and 98 were females, aged 39–85 years old, with an average age of (40.21 ± 7.15) years old. Inclusion criteria: (1) according to the patient's clinical manifestations and physical signs, it is clearly diagnosed as CA; (2) all patients have indications for carbon dioxide laser and ALA photodynamic therapy; (3) the treatment and research methods to the patient were explained, and the patient's consent has been obtained. Exclusion criteria: (1) patients with other severe skin and venereal diseases; (2) patients with severe infection and immune dysfunction; (3) patients with severe heart, lung, liver, and kidney dysfunction. Randomized grouping table was used to divide into intervention group (125 cases) and conventional group (86 cases). There was no significant difference in gender, age, course of disease, and type of condyloma between the intervention group and the routine group (*P* > 0.05), as shown in Table 1.

### 2.2. Methods

The following data were collected from all patients: gender, age, smoking, drinking, diabetes, and hypertension. Patients in the conventional group were treated with carbon dioxide laser, the skin of patients was routinely disinfected, lidocaine gel was applied to the wart and its surroundings for infiltration anesthesia, and a carbon dioxide laser treatment device was used to adjust the power of the carbon dioxide laser according to the size, location, and scope of the patient's wart to perform laser resection of the wart. It is ensured that the resection range is 0.3 cm outside the wart lesion. After the resection of the lesion is completed, mupirocin ointment is applied on the surface of the excised skin lesion 1∼2 times/d for continuous treatment for 1 week. Patients in the intervention group were treated with carbon dioxide laser combined with ALA photodynamic therapy. The CO_2_ laser treatment method is the same as the conventional group, after 3 hours of carbon dioxide laser treatment, and ALA photodynamic therapy was performed. 5-Aminolevulinic acid solution was diluted with physiological saline to a concentration of 20%, and the diluted solution was applied to the wound with a disinfectant dressing for 3∼4 h. The photodynamic therapy instrument is used, and the treatment power is adjusted to 100 mW/cm^2^ and continuously treated for 20 minutes. The treatment is performed once a week and 4 consecutive treatments.

### 2.3. Indicators of Observation

Efficacy evaluation: the patients were followed up for 6 months after treatment, and the patients were judged according to their lesion improvement and recurrence. Significantly effective: the patient's wart lesions were reduced >95%, and no recurrence occurred. Effective: the area of the patient's warts is reduced by 50%–95%, and no new warts appear. Invalid: the area of the patient's warts is reduced by <50%, and new warts appear. Effective rate = (number of cases with remarkable effect + effective effect)/total number of cases × 100%. According to the efficacy of patients, all patients were divided into an effective group (markedly effective + effective) and an ineffective group. Adverse reactions: after treatment, the two groups of patients were followed up for 6 months, and the incidence of burning sensation, redness and pain, scars, ulcers, and other adverse reactions were counted and compared between the two groups.

### 2.4. Statistical Methods

The results of this experiment were statistically analyzed by SPSS 20.0 (SPSS Co., Ltd., Chicago, USA). Count data were expressed by (rate), and chi-square test was used for their comparison between groups. Measurement data were expressed by (mean ± standard deviation), and *t*-test was used for their comparison between groups. Multivariate analysis adopts the multiple logistic regression model. *P* < 0.05 indicates that the difference is statistically significant.

## 3. Results

### 3.1. Comparison of the Efficacy of the Two Groups

In the intervention group, 95 cases were markedly effective, 25 cases were effective, and 5 cases were ineffective. The total effective rate of treatment was 96.00% (as shown in Figure 1); in the conventional treatment group, 49 cases were markedly effective, 24 cases were effective, and 13 cases were ineffective. The total effective rate of treatment was 84.88%. The curative effect of the intervention group was significantly higher than that of the conventional group, and the difference was statistically significant (*χ*^2^ = 4.95, *P* < 0.05).

### 3.2. Comparison of the Incidence of Adverse Reactions

The total incidence of adverse reactions in the intervention group (8.00%) was lower than that in the conventional group (32.56%) (*P* < 0.05) as shown in Table 2.

### 3.3. Single Factor Analysis Affecting the Short-Term Prognosis of Patients with Condyloma Acuminatum

Univariate analysis showed that the patient's smoking history, drinking history, course of disease, wart area, and number of sexual partners were related to the short-term prognosis (*P* < 0.05) as shown in Table 3.

### 3.4. Analysis of Multiple Factors Affecting the Prognosis of Condyloma Acuminatum Patients

Multivariate logistic regression analysis showed that the patient's course of disease, the area of the wart body, and the number of sexual partners were independent factors affecting the prognosis of patients with condyloma acuminatum (*P* < 0.05) as shown in Tables 4 and 5.

## 4. Discussion

CA is caused by human papillomavirus infection [7, 8]. It often occurs in the anus and external genitalia. The size of warts, HPV infection, and frequency of recurrence are all related to the immune function of the body. CA tends to recur after treatment, and some patients persist in unhealing, which has a serious impact on the patient's physiology and psychology [9, 10].

There are many treatment methods for CA. The clinically effective treatments include laser, high-frequency electrosurgical, cryotherapy, and photodynamic therapy [11, 12]. Burning, freezing, and other methods are the main methods to eliminate condyloma acuminatum. Carbon dioxide laser uses high-power laser thermal effect to burn the wart. It is a common method for clinical treatment of CA. It can accurately and completely cut and destroy the wart [13, 14]. However, studies have pointed out that human papillomavirus infections can occur within 1 cm of the wart body of CA. The area of carbon dioxide laser resection of the wart body is mostly 0.3 cm in the wart body lesion. After the resection, there are more virus residues, which may cause postoperative recurrence and affect the efficacy [15, 16]. CA can also be surgically removed. However, most patients need to be hospitalized for surgery under spinal anesthesia. The wart has a rich blood supply and bleeding, and the wound is prone to infection. The abovementioned treatments are painful and often induce the occurrence of scars.

ALA photodynamic therapy uses photosensitizer and photodynamic principles, 5-aminolevulinic acid solution is wet applied around the wart body as a photosensitizer, and a photodynamic therapy device is used to achieve the purpose of targeted therapy, so as to kill the viruses and promote the apoptosis and necrosis of the tissues infected by warts virus [17, 18]. The results of this study concluded that the treatment of CA with carbon dioxide laser combined with ALA photodynamic therapy can improve the treatment effect of patients (*P* < 0.05). ALA photodynamic therapy can improve the killing effect on residual virus, promote the apoptosis of human papillomavirus infected tissue, and then improve the clinical efficacy [19]. The incidence of adverse reactions in the intervention group was lower than that in the conventional group (*P* < 0.05). Therefore, the carbon dioxide laser combined with ALA photodynamic treatment of CA treatment safety is high.

The univariate analysis of this study showed that the patient's smoking history, drinking history, course of disease, wart area, and number of sexual partners are related to the short-term prognosis. Multivariate logistic regression analysis showed that the patient's course of disease, the area of the wart body, and the number of sexual partners were independent factors affecting the prognosis of patients with CA. Analysis of the reasons is that the large area of the wart suggests that the patient's symptoms are more serious, and the surrounding infection area is increased, and the light spot area required for photodynamic therapy is also larger, resulting in insufficient response energy for photodynamic therapy, which affects the prognosis. Patients with more sexual partners often have the characteristics of excessive sex life and unclean sex life, which can easily lead to secondary damage to the mucosa of the skin lesions, and secondary infections lead to recurrence, which affects the prognosis. Therefore, for patients with larger warts, multiple irradiation units can be selected to ensure a better treatment effect. And, active sexual behavior education is provided to patients, sexual life must be tried to avoid during treatment, and protective measures must be taken.

In summary, the treatment of CA with the carbon dioxide laser combined with ALA photodynamic therapy can significantly improve the clinical efficacy, without increasing the incidence of related adverse reactions, and has important clinical therapeutic value. The course of the disease, the area of the wart, and the number of sexual partners are independent factors affecting the prognosis of patients with CA.

## Figures and Tables

**Figure 1:** Efficacy of the carbon dioxide laser combined with ELLA photodynamics in the treatment of condyloma acuminatum. The picture shows representative pictures of the treatment of patients with condyloma acuminatum by the carbon dioxide laser combined with ALA photodynamics.

**Table 1:** Clinical data of the two groups.

Group	*n*	Male/female (*n*)	Age (year)	Course of disease (month)	Types of condyloma acuminatum (*n*)			
					Papillary	Miliary	Cauliflower	Hybrid
Intervention group	125	70/55	41.60 ± 7.21	5.43 ± 1.30	44	20	30	31
Conventional group	86	43/43	39.80 ± 7.12	5.71 ± 1.64	30	21	9	26
*χ* ^2^/*t*	—	0.289	0.265	0.201	0.748			
*P*	—	0.497	0.845	0.325	0.719			

**Table 2:** Comparison of the incidence of adverse reactions between the two groups (*n*, %).

Group	*n*	Burning sensation	Redness and pain	Scar	Ulcer	Total incidence of adverse reactions
Intervention group	125	5 (4.00)	5 (4.00)	0 (0.00)	0 (0.00)	10 (8.00)
Conventional group	86	6 (6.98)	10 (11.62)	6 (6.98)	6 (6.98)	28 (32.56)
*χ* ^2^/*t*	—	—	—	—	—	17.768
*P*	—	—	—	—	—	<0.001

**Table 3:** Single factor analysis affecting the prognosis of patients with condyloma acuminatum.

Factors	*n*	Effective group (*n* = 193)	Ineffective group (*n* = 18)	*χ* ^*2*^	*P*
Gender	—	—	—	0.657	0.418
Male	113	105 (54.40)	8 (44.44)	—	—
Female	98	88 (45.60)	10 (55.56)	—	—
Age (years)	—	—	—	0.571	0.449
≥60	100	93 (48.19)	7 (38.89)	—	—
<60	111	100 (51.81)	11 (61.11)	—	—
Smoking history	—	—	—	4.238	0.039
Yes	128	113 (58.55)	15 (83.33)	—	—
No	83	80 (41.45)	3 (16.67)	—	—
Drinking history	—	—	—	4.642	0.031
Yes	113	99 (51.30)	14 (77.78)	—	—
No	98	94 (48.70)	4 (22.22)	—	—
Course of disease (months)	—	—	—	5.694	0.017
≤1	126	120 (62.18)	6 (33.33)	—	—
>1	85	73 (37.82)	12 (66.67)	—	—
Wart body area (cm^2^)	—	—	—	5.824	0.016
<1.5	79	77 (39.90)	2 (11.11)	—	—
≥1.5	132	116 (60.10)	16 (88.89)	—	—
Number of sexual partners	—	—	—	7.778	0.005
<3	153	145 (75.13)	8 (44.44)	—	—
≥3	58	48 (24.87)	10 (55.56)	—	—

**Table 4:** Assignment for multivariate analysis of factors.

Factors	Variable	Assignment
Smoking history	X1	No = 0, yes = 1
Drinking history	X2	No = 0, yes = 1
Course of disease	X3	≤1 = 0, >1 = 1
Wart body area	X4	<1.5 = 0, ≥1.5 = 1
Number of sexual partners	X5	<3 = 0, ≥3 = 1

**Table 5:** Analysis of multiple factors affecting the short-term prognosis of condyloma acuminatum patients.

Variables	B	S.E	Wald's	*P*	OR	95% CI
Smoking history	1.035	1.984	1.608	0.181	2.815	0.746∼5.842
Drinking history	0.441	0.205	2.184	0.105	1.554	0.169∼4.057
Course of disease	1.102	0.564	5.015	0.025	3.011	1.408∼4.861
Wart body area	1.345	0.362	6.184	0.017	3.838	1.928∼5.908
Number of sexual partners	1.084	0.331	8.915	<0.001	2.956	1.625∼5.203

## Data Availability

The data used and/or analyzed during the current study are available from the corresponding author upon request.
